# Baicalein mediates inhibition of migration and invasiveness of skin carcinoma through Ezrin in A431 cells

This article has been retracted.

**DOI:** 10.1186/1471-2407-11-527

**Published:** 2011-12-28

**Authors:** Bin Wu, Ji Li, Damao Huang, Weiwei Wang, Yu Chen, Youxiang Liao, Xiaowei Tang, Hongfu Xie, Faqing Tang

**Affiliations:** 1 Department of Dermatology, Xiangnan College, Chenzhou 423000, P.R. China; 2 Department of Dermatology, Xiangya Hospital, Central South University, Changsha 410008, P.R. China; 3 Department of Clinical Laboratory, Xiangya Hospital, Central South University, Changsha 410008, P.R. China; 4 Metallurgical Science and Engineering, Central South University, Changsha 410008, P.R. China; 5 Department of Clinical Laboratory, Zhuhai Hospital, Jinan University, Zhuhai 519000, P.R. China

## Abstract

**Background:**

Ezrin is highly expressed in skin cancer and promotes tumor metastasis. Ezrin serves as a promising target for anti-metastasis therapy. The aim of this study is to determine if the flavonoid bacailein inhibits the metastasis of skin cancer cells through Ezrin.

**Methods:**

Cells from a cutaneous squamous carcinoma cell line, A431, were treated with baicalein at 0-60 μM to establish the non-cytotoxic concentration (NCC) range for baicalein. Following treatment with baicalein within this range, total Ezrin protein (both phosphorylated and unphosphorylated forms) and phosphorylated-Ezrin (phos-Ezrin) were detected by western blotting, and Ezrin RNA was detected in A431 cells using reverse transcription-polymerase chain reaction (RT-PCR). Thereafter, the motility and invasiveness of A431 cells following baicalein treatment were determined using wound-healing and Boyden chamber invasion assays. Short-interfering RNA (si-RNA) specifically targeting Ezrin was transfected into A431 cells, and a si-RNA Ezrin-A431 cell line was established by G418 selection. This stable cell line was transiently transfected with Ezrin and mutant Ezrin plasmids, and its motilityand invasiveness was subsequently determined to clarify whether bacailein inhibits these processes through Ezrin.

**Results:**

We determined the range of NCCs for baicalein to be 2.5-40 μM in A431 cells. Baicalein displayed a dose- and time-dependent inhibition of expressions of total Ezrin and phos-Ezrin within this range NCCs. In addition, it exerted this inhibitory effect through the reduction of Ezrin RNA transcript. Baicalein also inhibited the motility and invasiveness of A431 skin carcinoma cells within the range of NCCs, in a dose- and time-dependent manner. A431 cell motility and invasiveness were inhibited by 73% and 80% respectively when cells were treated with 20 μM baicalein. However, the motility and invasiveness of A431 cells containing the Ezrin mutant were not effectively inhibited by baicalein.

**Conclusions:**

Baicalein reduces the migration and invasiveness of A431 cells through the inhibition of Ezrin expression, which leads to the suppression of tumor metastasis.

## Background

Ezrin is a member of the ezrin-radixin-moesin (ERM) protein family that crosslinks the epithelial cell membrane with cytoskeleton. Ezrin helps maintain cell shape and motility, binds to adhesion molecules and participates in the regulation of intracellular signal transduction [1-4]. It is reported that Ezrin has an abnormal expression and a modified subcellular localization in tumor cells. Ezrin serves as a crosslinking molecule between the membranes of keratinocytes and cytoskeleton. Interacting with other adhesion molecules, Ezrin plays an essential part in the development of tumors, by promoting the proliferation and infiltration of tumor cells, metastasis, neovascularisation, and other biological mechanisms involved in malignancy [5-10]. In addition, Ezrin is considered an important potential anti-tumor drug target molecule [8-10].

One important mechanism for regulating the function of Ezrin is through phosphorylation of a conserved threonine residue in the C terminus of Ezrin protein (Thr-567) [11-14]. Non-phosphorylated Ezrin exists in a folded conformation, which results in the masking of its binding sites for other molecules. Phosphorylation at the conserved threonine residue causes conformational changes in Ezrin, unmasking its binding sites [11,14]. Phosphorylation of Ezrin at Thr 567 keeps it open and active, and prolongs its half-life [11]. Phosphorylated-Ezrin (phos-Ezrin) may be involved in various functions, including cell adhesion and motility, as well as the organization of cell surface structure.

Baicalein (5,6,7-trihydroxy-2-phenyl-4H-1-benzopyran-4-one) is one of four major flavanoids found in *Scutellaria baicalensis *Georgi, an herb widely used to treat various inflammatory diseases and ischemia [15]. In addition to its effectiveness against free radicals, baicalein has been reported to have a variety of other functions [16,17]. Recently, baicalein was discovered to have anti-cancer activity through inhibition of the Phosphoinositide 3-kinase (PI3K) pathway [18]. It also exerts proapoptotic activity through reactive oxygen species (ROS)-mediated and Ca^2+^-dependent mitochondrial dysfunction pathways in various cell types [19]. Bacailein has an inhibitory effect on lung cancer [20], colorectal cancer [21], gastric cancer [22], ovarian cancer [23], breast cancer [24], prostate cancer, and skin cancer [25,26]. Baicalein was also shown to inhibit the Epstein-Barr virus (EBV) early antigen activation induced by 12-O-tetradecanoylphorbol-13-acetate, and inhibit mouse skin tumors in an *in vivo *two-stage carcinogenesis model [27]. In particular, it was found that its anti-tumor effects in skin cancer were associated with inhibition of the p12-LOX pathway [28]. However, little is known about the molecular mechanisms of its anti-metastatic effects. Here, we show a novel anti-metastatic mechanism for baicalein in skin cancer cells, through inhibition of Ezrin and phos-Ezrin in A431 cells.

## Methods

### Reagents and antibodies

Chemical reagents, including dimethyl sulfoxide (DMSO), Tris, HCl, sodium dodecyl sulfate, and MTT [3-(4,5-dimethylthiazol-2-yl)-5-(3-carboxyme-thoxyphenyl)-2-(4-ulfophenyl)-2H-tetrazolium] were purchased from Sigma-Aldrich (St.Louis, MO). Baicalein was purchased from Sigma-Aldrich (St.Louis, MO), and stored at 4°C under dark conditions. The stock solution of baicalein for incubation with cells was prepared in DMSO and further diluted in the culture medium. The final DMSO concentration in the medium was 0.1% (in control or treated samples), which did not affect cell viability. TRIozl reagent was purchased from Invitrogen. Antibody against Ezrin was purchased from Covance (Berkeley, CA), antibody against phosphorylated Ezrin at Thr-567 (phos-Ezrin Thr-567) was purchased from Cell Signaling Technology (Danvers, MA) and antibodies against β-actin and normal mouse immunoglobulin G (IgG) were purchased from Santa Cruz Biotechnology, Inc. (Santa Cruz, CA). The secondary antibodies horseradish peroxidase-linked anti-mouse IgG and anti-rabbit IgG were purchased from Santa Cruz Biotechnology, Inc. The protein assay kit was purchased from Bio-Rad (Herndon, VA).

### Cell culture and baicalein treatment

A431 cells (human squamous carcinoma cell line) were purchased from the Shanghai Cell Biological Institute of the Chinese Academy of Science (Shanghai 200007, China). The cell line was cultured as a monolayer in RPMI-1640 medium containing 10% fetal bovine serum, 2 mM L-glutamine, 100 μg/ml penicillin, 100 mg/ml streptomycin (Invitrogen, Carlsbas, CA), and maintained in an incubator with a humidified atmosphere of 95% air and 5% CO_2 _at 37°C. For baicalein treatment, appropriate amounts of stock solution of baicalein were added to the cultured cells to achieve the indicated concentrations and then incubated for the indicated time points. Following baicalein treatment, cell viability was determined using MTT assays. To determine if baicalein inhibited Ezrin and phos-Ezrin in a dose-dependent manner, A431 cells were treated with 10, 20, and 40 μM baicalein for 24 h. To determine if baicalein inhibited Ezrin and phos-Ezrin in a time-dependent manner, A431 cells were treated with 20 μM baicalein for 24, 48, and 72 h. After treatment with baicalein, the cells were harvested, and proteins were extracted from the cell samples. Expressions of Ezrin and phos-Ezrin were detected by western blotting.

### Determination of cell viability (MTT assay)

To evaluate the cytotoxicity of baicalein, MTT assays were performed to determine cell viability. A431 cells were seeded in 96-well plates at a density of 3.5 × 10^3 ^cells/well and treated with baicalein at 0-60 μM concentrations at 37°C for 48 h. After the exposure period, cell media was removed, and cells were washed with phosphate-buffered saline (PBS). Thereafter, the media was changed and cells were incubated with 100 μl MTT (5 mg/ml) for 4 h. The total number of viable cells per dish is directly proportional to the production of formazan, which was solubilized in isopropanol, and measured spectrophotometrically at 563 nm [29].

### Western blotting analysis

After treatment with baicalein, cell samples were disrupted with 0.6 ml lysis buffer (1 × PBS, 1% Nonidet P-40, 0.5% sodium deoxycholate, 0.1% sodium dodecyl sulfate, 100 μg/ml phenylmethanesulfonyl fluoride, 10 μg/ml aprotinin, and 1 mM sodium orthovanadate). The cell lysate was then subjected to a centrifugation of 10,000× *g *for 10 min at 4°C. The supernatant protein concentration of each sample was determined using the Bio-Rad Protein Assay (Bio-Rad Laboratories, Inc., Hercules, CA). Protein (40 μg) from each sample was separated using a 10% polyacrylamide gel and transferred onto a nitrocellulose membrane. The blot was subsequently incubated with 5% non-fat milk in PBS for 1 h to block non-specific binding, and incubated with specific antibodies against Ezrin (Covance) or phos-Ezrin (Cell Signaling Technology) for 2 h and incubated with an appropriate peroxidase-conjugated secondary antibody (Sigma, St. Louis, MO) for 1 h. All incubations were carried out at 37°C. The blot was washed 3 times in PBS, and the signal was developed using 4-chloro-1-napthol/3,3-o-diaminobenzidine. The relative photographic density was quantified by scanning the photographic negative using a gel documentation and analysis system. β-actin was used as an internal control to verify basal protein expression levels of Ezrin and phos-Ezrin, as well as equal protein loading.

### RT-PCR for detecting Ezrin RNA

To detect Ezrin RNA in A431 cells following baicalein treatment, we performed reverse transcription-polymerase chain reaction (RT-PCR). A431 cells were initially treated with baicalein at various concentrations (5, 10, 20, and 40 μM) for 48 h. The cell samples were then harvested, and RNAs in these samples were extracted using TRIozl and following the manufacturer's suggested protocol (Invitrogen). For detecting Ezrin RNA, primers for PCR were designed based on GenBank sequences for full-length human Ezrin and β-actin cDNA. The following primer sequences were used: for ezrin, primer 1 (sense) 5'-CTCATCCAGGACATCACCCA-3', primer2 (antisense) 5'-TCACTCCAAGGAAAG CCAAT 3'. The corresponding PCR product was 450 bp. For β-actin, primer 3 (sense), 5'-GACAGGATGCAGAAGGAGAT-3', primer2 (antisense) 5'-TGTGTGGACTTGGGAG AGGACT-3'. The corresponding PCR product was 550 bp. The PCR products were visualized using agarose gel electrophoresis. Following electrophoresis, the relative PCR product band densities were quantified by densitometry using ImageQuant image analysis system (Storm Optical Scanner, Molecular Dynamics). β-actin was used as an internal control to verify the basal expression level of Ezrin and equal RNA loading.

### Wound-healing assays

A431 and si-RNA Ezrin-A341 cells (2 × 10^6^) were seeded in 10-mm plates at 37°C for 24 h. Confluent monolayer of A431 was then wounded using a plastic tip. Cells were treated with baicalein at 20 μM, and then photographed after 48 h. Cells moving cross the boundaries lines were counted.

### Cell invasion and motility assay

For cell invasion assay, A431 cells were treated with different concentrations of baicalein. After 24 h of treatment, cells were removed by trypsinization, and their invasiveness was tested *in vitro *using a Boyden chamber invasion assay [30]. Matrigel (Collaborative Biomedical Products, Bedford, MA) was diluted to 0.5 mg/ml with cold filtered distilled water and applied to 8-mm pore size polycarbonate membrane filters. Treated cells were seeded in a Boyden chamber (Neuro Probe, Cabin John, MD) at a density of 1.5 × 10^4 ^cells/well in 50 μl of serum-free-medium in the top well of the chamber and then incubated for 12 h at 37°C. The bottom well contained standard medium with 20% fetal bovine serum. The cells that invaded the lower surface of the membrane were fixed with methanol and stained with hematoxylin and eosin. Random fields were counted for cells that had invaded the membrane, using an optics microscope. To determine the effect of baicalein on cell motility, cells were seeded in a Boyden Chamber on membrane filters, which were not coated with Matrigel. The motility of cells treated or untreated with baicalein was measured as previously described [30]. The statistical analysis was corrected for cell viability to clarify the effect of baicalein.

### Construction of expression vectors

A full-length Ezrin DNA fragment was generated by PCR and subcloned into a pcDNA3.1 vector (Amersham Biosciences Corp., Piscataway) to generate a pcDNA3.1-Ezrin plasmid [29]. A plasmid containing a mutant form of Ezrin (pcDNA3.1-Ezrin M) was generated with the QuickChange II site-directed mutagenesis kit and Ezrin mutant primers: Primer 1 (sense), 5'-CAGGGCAACGCCAAGCAGCGCAT-3'; Primer 2 (antisense), 5'-ATGCGCTGCTTGGCGTTGCCCTG-3' (Thr567 was muted into Ala 567). The pU6pro vector was used to construct a non-specific control vector containing a scrambled sequence (si-mock), as well as two si-RNA vectors specifically targeting Ezrin (si-Ezrin). The pU6pro-si-mock and pU6pro-si-Ezrin vectors were generated following the manufacturer's recommended protocol. Primers were synthesized for si-mock (general scramble: sense, 5'-TTTGACTACCGTTGTTATAGGTGTTCAAGAGACACC TATAACAACGGTAGTTTTTT-3'; antisense, 5'-CTAGAAAAAACTACCGTTGTTAT AGGTGTCTCTTGAACACCTATAACAACGGTAGT-3') and si-Ezrin (Set 1, 5'-CCCCAAAGATTGG CTTTCC-3' (position in the open reading frame, 704-722); Set 2, 5'-TCCACTATGTGGATAATAA-3' (open reading frame, 140-158) (Ambion, Texas) [29]. All constructs were confirmed by restriction enzyme mapping and DNA sequencing.

### Generation of stable cell lines

A431 cells (5.0 × 10^5^) were transfected with pU6pro-si-Ezrin constructs using Lipofectamine2000 reagent (Life Technologies, Inc.) following the manufacturer's suggested protocol. si-RNA Ezrin-A341 stably-transfected cell lines were obtained by selection for G418 resistance (400 μg/ml). Ezrin knockdown was confirmed by assessing Ezrin expression. si-RNA Ezrin-A341 cell lines were transiently transfected with 4 μg of pcDNA3.1, pcDNA3.1-Ezrin, or pcDNA3.1-Ezrin M. After baicalein treatment, the invasion and motility of these stably-transfected cell lines were determined using a Boyden chamber invasion assay.

### Statistical analysis

Each assay was performed in triplicate. Data are expressed as the mean ± standard deviation (SD). The statistical significance of the data obtained were evaluated using the Student's *t*-test (* *p *< 0.05).

## Results

### Cytotoxicity assay for baicalein in skin cancer cells

Baicalein is a flavonoid found in *Scutellaria baicalensis *Georgi, which is the aglycone compound of baicaline. Its chemical structure is showed in Figure 1a. In this study, we determined the cytotoxicity of baicalein by treating A431 cells with various concentrations of baicalein for 48 h. Compared with the control treatment (0.1% DMSO), the cell viability of the samples treated with baicalein at concentrations between 2.5-40 μM was not significantly altered (Figure 1b), indicating that baicalein was not cytotoxic to A431 cells at these dosages. Hence, 2.5-40 μM was determined to be a range of the non-cytotoxic concentration (NCC) of bacailein on A431 cells. This range of concentrations was therefore applied in all subsequent experiments.

**Figure 1:** **Effect of baicalein on the viability of A431 cells**. a. Structure of baicalein, which is the aglycone compound of baicaline. b. A431 cells were treated with 0, 2.5, 5, 10, 20, 40, 50, or 60 μM of baicalein for 48 h before being subjected to an MTT assay for cell viability. Data were represented as the mean ± SD from three independent experiments. Baicalein had no cytotoxic effect on A431 cells at a range of 2.5-40 μM. Results were statistically analyzed with a Student's t-test (*p < 0.05). The error bars represent SDs.

### Suppression of Ezrin expression by baicalein

To determine if baicalein had an inhibitory effect on Ezrin, a NCC of baicalein (10-40 μM) was used to treat A431 cells, and then total Ezrin and phos-Ezrin expression levels were detected with western blotting. After baicalein treatment, total Ezrin and phos-Ezrin expression levels dramatically decreased compared with the control (Figure 2a, lane 1 *vs *2, 3, 4 in the upper and middle panels), and this decrease was dose-dependent. To determine if this inhibition was dependent on the length of time, 20 μM baicalein was used to treat A431 cells for 12, 24, and 48 h, and total Ezrin and phos-Ezrin expression levels were examined. The results suggest that the inhibitory effect of baicalein on total Ezrin and phos-Ezrin was time-dependent (Figure 2b, lane 1 *vs *2, 3, 4 in the upper and middle panels). To determine if the inhibitory effect of baicalein on Ezrin protein expression occurs through downregulation of Ezrin RNA, Ezrin RNA expression was detected in A431 cells treated with baicalein using RT-PCR. Following baicalein treatment, Ezrin RNA expression dramatically decreased in a dose-dependent manner (Figure 3a, lane 2 *vs *3, 4, 5, 6, and Figure 3b, lane 1 *vs*. 2, 3, 4, 5).

**Figure 2:** **The inhibitory effects of baicalein on Ezrin and phos-Ezrin in A431 cells**. a. A431 cells were treated with baicalein at 0, 10, 20, and 40 μM for 24 h. b. A431 cells were treated with 20 μM baicalein for 12, 24, and 48 h. After baicalein treatment, total protein was extracted from these cell samples. The protein samples were then subjected to western blotting, and the levels of Ezrin and phos-Ezrin expression in these samples were determined. Baicalein inhibited the expression of Ezrin and phos-Ezrin at Thr-567 in a dose- and time-dependent manner. β-actin or Ezrin respectively served as the control for quantifying Ezrin or phos-Ezrin. Three independent experiments were carried out and representative figures are shown.

**Figure 3:** **Inhibitory effect of baicalein on Ezrin RNA in A431 cells**. A431 cells were treated with baicalein at 0, 5, 10, 20, and 40 μM for 48 h. After baicalein treatment, the cell samples were harvested, and RNAs in these samples were extracted. Ezrin RNA expression was detected by RT-PCR. 0.1% DMSO served as the blank control. β-actin served as the loading control. The expression of Ezrin RNA in A431 cells gradually decreased with increasing baicalein concentrations. Three independent experiments were carried out and representative figures are shown.

### Inhibitory effect of baicalein on the motility and invasiveness of A431 cells

Ezrin is associated with cell motility in tumor invasion. As a first step towards examining the effect of baicalein on Ezrin expression and function, we investigated whether baicalein could inhibit the invasion and motility of A431 cells *in vitro*. We used wound-healing assays to test the migration of A431 cells with baicalein treatment. Following baicalein treatment, the motility of A431 cells was significantly inhibited, and consequently the cells were unable to migrate into the wound (Figure 4, panel a *vs*. b and lane 1 *vs*. 2 in panel c, *p < 0.05). Same as Figure 4-(b), the crawling movement of cells was also inhibited when transfected with Ezrin si-RNA (Figure 4-c). Ezrin expression dramatically decreased following baicalein treatment and Ezrin si-RNA transfection (Figure 4-e). There were virtually no scratches across the boundaries and the migration of A431 cells was not observed. Hence, we concluded that there was no significant difference in the migration of Ezrin si-RNA transfected cells and cells treated with baicalein.

**Figure 4:** **Inhibitory effects of baicalein on A431 cell migration**. A431 cells (2 × 10^6^) were seeded in 10-mm plates and incubated at 37°C for 48 h. Confluent monolayers of A431 cells were then wounded using a plastic tip. The cells were treated with 20 μM baicalein, then photographed after 48 h. The cells migrating cross the boundaries lines in the center of the wells were counted, and Ezrin expression was examined in the cell samples. (a) A431 cells treated with 0.1% DMSO. (b) A431 cells treated with 20 μM baicalein. (c) A431 cells transfected with Ezrin si-RNA. (d) Numbers of cells that moved cross the lines (10 fields). (e) Ezrin expression in A431 cells with 0.1% DMSO, 20 μM baicalein or Ezrin si-RNA, respectively. The data are represented as the mean ± SD from three independent experiments. Results were statistically analyzed using one-way analysis of variance (ANOVA) with a post hoc Dunnett's test (* *p *< 0.05). The error bars represent SDs.

To examine the invasiveness of A431 cells following baicalein treatment, a Boyden chamber coated with Matrigel was used. The results suggested that the number of cells that invaded the lower chamber was significantly reduced by baicalein treatment (Figure 5A-b; Figure 5A-c, lane 2 *p < 0.05). The observed reduction was concentration-dependent, with 80% inhibition occurring when 20 μM baicalein was used (Figure 5A-c). A similar inhibitory effect was also observed for the mobility of baicalein-treated cells. To further test the time and dose-dependence of the inhibitory effects observed, A431 cells were treated with baicalein at various concentrations or time points, and then subjected to analyses for motility and invasiveness. After baicalein treatment, the motility and invasive abilities of cells were decreased in a dose-dependent manner, there was only 27% mobility and 21% invasion when cells were treated with 20 μM baicalein, and 16% motility and in 11% invasion when treated with 40 μM baicalein (Figure 5B, C, *p < 0.05). The cells also displayed a time-dependent reduction in these properties (Figure 5D, E, *p < 0.05, **p < 0.01). Hence, these results indicated that baicalein could inhibit A431 cell migration and invasiveness in a dose and time-dependent manner.

**Figure 5:** **Inhibitory effects of baicalein on the motility and invasiveness of A431 cells**. A431 cells were treated with 20 μM bacailein, and cell invasiveness was detected using Boyden Chamber with Matrigel coating. A-(a), Invasiveness of control cells (treated with 0.1% DMSO). A-(b), Invasiveness of cells treated with 20 μM baicalein. Scale bar, 10 μm. A-(c), Numbers of cells invading through the filters of chamber (10 fields). To test for dose-dependence, A431 cells were treated with baicalein at 20 or 40 μM for 48 h, and for the time-course experiment, A431 cells were treated with 20 μM baicalein for 24, 48, and 72 h. The cells were then subjected to analyses for motility and invasion abilities as described in Methods. B. Motility of A431 cells at various concentrations of baicalein. C. Invasiveness of A431 cells at various concentrations of baicalein. D. Motility of A431 cells at various time points. E. Invasion of A431 cells at various time points. The data are represented as the mean ± SD from three independent experiments. Results were statistically analyzed using one-way ANOVA with post hoc Dunnett's *test *(* *p *< 0.05). The error bars represent SDs. IR, invasion rate. MR, motility rate.

### Suppression of the migration and invasiveness of A431 cells by baicalein through Ezrin

To test if the reduction of motility and invasiveness of A431 cells by baicalein occurs through Ezrin, si-RNA targeting Ezrin was transfected into A431 cells. si-RNA Ezrin-A431 cells were then transiently transfected with pcDNA3.1, pcDNA3.1-Ezrin M or pcDNA3.1-Ezrin and then treated with 20 μM baicalein for 48 h. The motility and invasiveness of the cells were then evaluated. Following baicalein treatment, the invasiveness and motility of cells transfected with pcDNA3.1-Ezrin dramatically decreased compared with the control-transfected cells (Figure 6b, lane 5 *vs*. 6, and Figure 6c, lane 5 *vs*. 6, *p < 0.01). Ezrin expression was also decreased compared with control cells (Figure 6a, lane 5 *vs*. 6 in the upper panel). si-RNA Ezrin-A431 cells transfected with pcDNA3.1-Ezrin M did not show decreased motility and invasiveness (Figure 6b, lane 3 *vs*. 4, and Figure 6c, lane 3 *vs*. 4). In the transfects with pcDNA3.1-Ezrin M, Ezrin expression decreased when baicalein treatment (Figure 6a, lane 3 *vs*. 4), and baicalein degraded Ezrin expression, but the motility and invasion of cells did not alter (Figure 6b, lane 3 *vs*. 4, and Figure 6c, lane 3 *vs*. 4). These data suggest that baicalein inhibits Ezrin expression, and consequently decreases the invasiveness and migration of skin cancer cells.

**Figure 6:** **Suppression of motility and invasiveness of A431 cells by baicalein through Ezrin**. si-RNA Ezrin-A431 cells were transiently transfected with pcDNA3.1, pcDNA3.1-Ezrin M, or pcDNA-Ezrin and then treated with bacailein. a. Ezrin expression in the transfected cells was detected by western blotting. β-actin served as a loading control. The transfected cells were then subjected to analyses for motility (b) and invasion (c) as described in Methods. Data are represented as the mean ± SD from three independent experiments. Results were statistically analyzed using one-way ANOVA with post hoc Dunnett's *test *(* p < 0.05). The error bars represent SDs.

## Discussion

Ezrin is overexpressed in a variety of neoplastic cells including skin cancers [31], and is involved in the later stages of tumor progression and metastasis. It is expressed in most primary melanomas of the skin and in all metastatic tumors. Ezrin expression correlates with tumor thickness and level of invasion, which suggests an association between Ezrin expression and tumor progression [32]. The intensity of Ezrin immunoreactivity was found to increase with tumor size, as measured by tumor thickness (Breslow classification) and invasion to dermal layers (Clark classification) [33]. The assessment of Ezrin expression may be exploited as a new tool to evaluate the malignancy of human melanoma. In addition, gene therapy or drug treatments aimed at inhibiting actin assembly to the phagosomal membranes may be proposed as a new strategy for the control of tumor aggressiveness [34].

Baicalein, a major flavonoid from a traditional Chinese herb *Scutellaria baicalensis *Georgi (Huangqin), which is the aglycone compound of baicaline, possesses potent anti-cancer properties. It has been reported that baicalein inhibited mouse skin tumors in an *in vivo *two-stage carcinogenesis model [27]. Pretreatment of mouse skin with various amounts of baicalein caused inhibition of H_2_O_2 _and myeloperoxidase formation by 12-O-tetradecanoylphorbol-13-acetate. These results indicate that baicalein serves as a potential cancer-chemopreventive agent against tumors [25]. In the present work, A431, a human epithelial carcinoma cell line with high malignancy and high expression of Ezrin, was used to investigate the inhibitory mechanism of baicalein. To distinguish anti-cancer effects from cytotoxicity to cells, we first measured the NCCs of baicalein that could be used on A431 cells. We determined 0-40 μM to be the range of NCCs that could be used. We next set out to test if baicalein had an inhibitory effect on Ezrin. We found that Ezrin expression was effectively inhibited by baicalein. In addition, Ezrin function was previously reported to be regulated by phosphorylation of Thr-567 at its C-terminus [11-14]. We found that baicalein could effectively inhibit the phosphorylation of Ezrin at Thr-567 of C terminus. Furthermore, baicalein exerted its inhibitory effect by suppressing the Ezrin RNA transcript. Based on the above results, we believe that baicalein specifically inhibits Ezrin expression and phosphorylation.

Ezrin is involved in a variety of cellular functions, including cell adhesion, motility, and the organization of cell surface structure [3,4]. We speculate that baicalein represses Ezrin expression at RNA transcript, and reduces Ezrin and phos-Ezrin protein expression, inhibits cell migration and tumor invasion. Interestingly, baicalein had no effect on the motility and invasiveness of A431 cells transfected with a mutant form of Ezrin Ala 567. Although Baicalein also inhibited Ezrin expression in the transfect with pcDNA3.1-Ezrin M, baicalein may degrade Ezrin expression, the motility and invasion of cells did not alter after bacailein treatment. Baicalein may inhibit 6-10B cell migration and invasion mainly through reducing phos-Ezrin at Thr 567. These results indicate that baicalein mediates the reduction of migration and invasiveness of A431 cells through phos-Ezrin at Thr567. Baicalein may serves as a novel drug for skin cancer therapy in the future.

## Conclusion

Here, we provide evidence that baicalein inhibits the invasive abilities of skin cancers through Ezrin. Baicalein inhibits the migration and invasiveness of A431 cells, following the reduction of Ezrin, phos-Ezrin and Ezrin RNA. However, baicalein had no effect on A431 cells transfected with an Ezrin mutant at 567, suggesting that its inhibitory effect on cell migration and tumor invasiveness occurs mainly through phos-Ezrin at Thr 567.

## Competing interests

The authors declare that they have no competing interests.

## Authors' contributions

BW performed the NCC assay, cell culture and statistical analyses, and wrote the paper. JL performed RT-PCR, designed the PCR primers and controlled the quality of the PCR reactions. DMH constructed the plasmids and tested cell motility and invasion. WWW performed the western blots. YC performed the cell transfections and established the stable cell lines. XWT performed statistical analyses and revised the paper. HFX performed cell culture. FQT coordinated the study and revised the paper. All authors read and approved the final manuscript.

## Pre-publication history

The pre-publication history for this paper can be accessed here:

http://www.biomedcentral.com/1471-2407/11/527/prepub

## References

[B1] MiaczynskaMPelkmansLZerialMNot just a sink: endosomes in control of signal transductionCurr Opin Cell Biol200416440040610.1016/j.ceb.2004.06.00515261672

[B2] GouldKLBretscherAEschFSHunterTcDNA cloning and sequencing of the protein-tyrosine kinase substrate, ezrin, reveals homology to band 4.1Embo J198981341334142259137110.1002/j.1460-2075.1989.tb08598.xPMC401598

[B3] SaotomeICurtoMMcClatcheyAIEzrin is essential for epithelial organization and villus morphogenesis in the developing intestineDev Cell20046685586410.1016/j.devcel.2004.05.00715177033

[B4] FaureSSalazar-FontanaLISemichonMTybulewiczVLBismuthGTrautmannAGermainRNDelonJERM proteins regulate cytoskeleton relaxation promoting T cell-APC conjugationNat Immunol20045327227910.1038/ni103914758359

[B5] PalouJAlgabaFVeraIRodriguezOVillavicencioHSanchez-CarbayoMProtein Expression Patterns of Ezrin Are Predictors of Progression in T1G3 Bladder Tumours Treated with Nonmaintenance Bacillus Calmette-GuerinEur Urol200956582983610.1016/j.eururo.2008.09.06218926620

[B6] KocherHMSandleJMirzaTALiNFHartIREzrin interacts with Cortactin to form podosomal rosettes in pancreatic cancer cellsGut200958227128410.1136/gut.2008.15987118852256

[B7] WangGMaoWZhengSMicroRNA-183 regulates Ezrin expression in lung cancer cellsFEBS Lett200858225-263663366810.1016/j.febslet.2008.09.05118840437

[B8] ElzagheidAKorkeilaEBendardafRBuhmeidaAHeikkilaSVaheriASyrjanenKPyrhonenSCarpenOIntense cytoplasmic ezrin immunoreactivity predicts poor survival in colorectal cancerHum Pathol200839121739174310.1016/j.humpath.2008.04.02018701134

[B9] LiQWuMWangHXuGZhuTZhangYLiuPSongAGangCHanZEzrin silencing by small hairpin RNA reverses metastatic behaviors of human breast cancer cellsCancer Lett20082611556310.1016/j.canlet.2007.11.01818155831

[B10] PengSFanSLiXWangLLiuHZhouMShenSLiGThe expression of ezrin in NPC and its interaction with NGX6, a novel candidate suppressorCancer Sci200798334134910.1111/j.1349-7006.2007.00410.x17270023PMC11158500

[B11] MatsuiTMaedaMDoiYYonemuraSAmanoMKaibuchiKTsukitaSRho-kinase phosphorylates COOH-terminal threonines of ezrin/radixin/moesin (ERM) proteins and regulates their head-to-tail associationJ Cell Biol1998140364765710.1083/jcb.140.3.6479456324PMC2140160

[B12] ChenJCohnJAMandelLJDephosphorylation of ezrin as an early event in renal microvillar breakdown and anoxic injuryProc Natl Acad Sci USA199592167495749910.1073/pnas.92.16.74957638219PMC41366

[B13] YonemuraSMatsuiTTsukitaSRho-dependent and -independent activation mechanisms of ezrin/radixin/moesin proteins: an essential role for polyphosphoinositides in vivoJ Cell Sci2002115Pt 12256925801204522710.1242/jcs.115.12.2569

[B14] ZhuLZhouRMettlerSWuTAbbasADelaneyJForteJGHigh turnover of ezrin T567 phosphorylation: conformation, activity, and cellular functionAm J Physiol Cell Physiol20072933C87488410.1152/ajpcell.00111.200717553936

[B15] KimYOLeemKParkJLeePAhnDKLeeBCParkHKSukKKimSYKimHCytoprotective effect of Scutellaria baicalensis in CA1 hippocampal neurons of rats after global cerebral ischemiaJ Ethnopharmacol2001772-318318810.1016/S0378-8741(01)00283-511535362

[B16] Li-WeberMNew therapeutic aspects of flavones: the anticancer properties of Scutellaria and its main active constituents Wogonin, Baicalein and BaicalinCancer Treat Rev2009351576810.1016/j.ctrv.2008.09.00519004559

[B17] TongWGDingXZAdrianTEThe mechanisms of lipoxygenase inhibitor-induced apoptosis in human breast cancer cellsBiochem Biophys Res Commun2002296494294810.1016/S0006-291X(02)02014-412200139

[B18] KongDYamazakiKYamoriTDiscovery of phosphatidylinositol 3-kinase inhibitory compounds from the Screening Committee of Anticancer Drugs (SCADS) libraryBiol Pharm Bull20103391600160410.1248/bpb.33.160020823581

[B19] PidgeonGPKandouzMMeramAHonnKVMechanisms controlling cell cycle arrest and induction of apoptosis after 12-lipoxygenase inhibition in prostate cancer cellsCancer Res20026292721272711980674

[B20] LeeHZLeungHWLaiMYWuCHBaicalein induced cell cycle arrest and apoptosis in human lung squamous carcinoma CH27 cellsAnticancer Res2005252A95996415868934

[B21] LeaMAIbehCDeutschJKHamidIdesBordesCInhibition of growth and induction of alkaline phosphatase in colon cancer cells by flavonols and flavonol glycosidesAnticancer Res20103093629363520944146

[B22] ChenFLWangXZLiJYYuJPHuangCYChenZX12-lipoxygenase induces apoptosis of human gastric cancer AGS cells via the ERK1/2 signal pathwayDig Dis Sci200853118118710.1007/s10620-007-9841-117522976

[B23] WeiXGuoWWuSWangLHuangPLiuJFangBOxidative stress in NSC-741909-induced apoptosis of cancer cellsJ Transl Med201083710.1186/1479-5876-8-3720398386PMC2873373

[B24] WangLLingYChenYLiCLFengFYouQDLuNGuoQLFlavonoid baicalein suppresses adhesion, migration and invasion of MDA-MB-231 human breast cancer cellsCancer Lett20102971424810.1016/j.canlet.2010.04.02220580866

[B25] LeeMJWangCJTsaiYYHwangJMLinWLTsengTHChuCYInhibitory effect of 12-O-tetradecanoylphorbol-13-acetate-caused tumor promotion in benzo[a]pyrene-initiated CD-1 mouse skin by baicaleinNutr Cancer199934218519110.1207/S15327914NC3402_910578486

[B26] TaniguchiHYoshidaTHorinakaMYasudaTGodaAEKonishiMWakadaMKataokaKYoshikawaTSakaiTBaicalein overcomes tumor necrosis factor-related apoptosis-inducing ligand resistance via two different cell-specific pathways in cancer cells but not in normal cellsCancer Res200868218918892710.1158/0008-5472.CAN-08-112018974136

[B27] TsujiiHYamadaTKajimotoTTanakaRTokudaHHasegawaJHamashimaYNodeMHybrids of 3alpha-methoxyserrat-14-en-21beta-ol (PJ-1) and 3beta-methoxyserrat-14-en-21beta-ol (PJ-2) and various anti-oxidants as cancer chemopreventive agentsEur J Med Chem20104562191219710.1016/j.ejmech.2010.01.05720153563

[B28] PiaoYSDuYCOshimaHJinJCNomuraMYoshimotoTOshimaMPlatelet-type 12-lipoxygenase accelerates tumor promotion of mouse epidermal cells through enhancement of cloning efficiencyCarcinogenesis20082924404471817425310.1093/carcin/bgm274

[B29] TangFWangDDuanCHuangDWuYChenYWangWXieCMengJWangLBerberine inhibits metastasis of nasopharyngeal carcinoma 5-8F cells by targeting Rho kinase-mediated Ezrin phosphorylation at threonine 567J Biol Chem200928440274562746610.1074/jbc.M109.03379519651779PMC2785675

[B30] AttigaFAFernandezPMWeeraratnaATManyakMJPatiernoSRInhibitors of prostaglandin synthesis inhibit human prostate tumor cell invasiveness and reduce the release of matrix metalloproteinasesCancer Res200060164629463710969817

[B31] BretscherAEdwardsKFehonRGERM proteins and merlin: integrators at the cell cortexNat Rev Mol Cell Biol20023858659910.1038/nrm88212154370

[B32] IlmonenSVaheriAAsko-SeljavaaraSCarpenOEzrin in primary cutaneous melanomaMod Pathol200518450351010.1038/modpathol.380030015475929

[B33] GeigerKDStoldtPSchloteWDerouicheAEzrin immunoreactivity is associated with increasing malignancy of astrocytic tumors but is absent in oligodendrogliomasAm J Pathol200015761785179310.1016/S0002-9440(10)64816-X11106550PMC1885782

[B34] LuginiLLozuponeFMatarresePFunaroCLucianiFMalorniWRivoltiniLCastelliCTinariAPirisAPotent phagocytic activity discriminates metastatic and primary human malignant melanomas: a key role of ezrinLab Invest200383111555156710.1097/01.LAB.0000098425.03006.4214615410

